# A Novel Curcumin-Based Drug Powder Inhalation Medicine for Chronic Obstructive Pulmonary Disease

**DOI:** 10.1155/2021/8001787

**Published:** 2021-11-29

**Authors:** Qin Shen, Yongjie Jiang, Jing Chen, Xueling Wang, Jiao Zheng

**Affiliations:** ^1^Department of Respiratory Medicine, Hunan Provincial People's Hospital (The First-Affiliated Hospital of Hunan Normal University), Changsha 410005, China; ^2^Department of Gynecology and Obstetrics, Zhengzhou Big Bridge Hospital, Zhengzhou 450000, China; ^3^Department of Respiratory Medicine Lung Function Room, Hunan Provincial People's Hospital (The First-Affiliated Hospital of Hunan Normal University), Changsha 410005, China; ^4^Drug Clinical Trial Institution Department, Hunan Provincial People's Hospital (The First-Affiliated Hospital of Hunan Normal University), Changsha 410005, China

## Abstract

The dry powder inhaler is a new form of drug delivery that is widely used as an alternative to traditional drug delivery methods, addressing the shortcomings of traditional drug delivery methods and obtaining better therapeutic results. This mode of delivery is also one of the most rational ways to treat pulmonary diseases such as chronic obstructive pulmonary disease (COPD). Curcumin, a natural polyphenol, has been shown to be effective in the treatment of COPD. In this study, different concentrations of curcumin ethanol solution were spray dried with mannitol as a carrier to obtain dry powder particles with different particle size distribution for the preparation of curcumin dry powder inhaler. The solubility and physicochemical properties were further characterized by differential scanning calorimetry (DSC), X-ray diffraction (XRD), and scanning electron microscopy. The characterization results showed that the product obtained in the experiment had reasonable particle size distribution and excellent solubility properties, which were positive for the treatment of COPD or other pulmonary diseases.

## 1. Introduction

Chronic obstructive pulmonary disease (COPD) is a not fully reversible chronic respiratory disease that progresses slowly and is characterized by obstructive ventilation patterns, often associated with smoke, air pollution, radiation, and viral infections, and can lead to severe chronic respiratory failure [1, 2]. It is often combined with other respiratory comorbidities, pulmonary diseases such as pneumonia, pulmonary cancer, and pulmonary fibrosis, which severely impair pulmonary function and quality of life in patients of all ages [3, 4]. For pulmonary diseases, clinical treatments commonly used include medication, radiation therapy, and surgery. With pulmonary drug therapy, the use of traditional delivery methods, such as oral, intravenous, or intramuscular injections, often results in widespread distribution of drugs throughout the body's tissues [5]. This mode of drug delivery often brings adverse effects [5–9]:

1. Wide distribution of the drug in normal tissues, resulting in reduced therapeutic efficiency in the lungs
2. Irreversible damage caused by the systemic distribution of toxic agents
3. Some insoluble drugs have low bioavailability and do not achieve good therapeutic effects after oral administration
4. Instability of multiple drugs in the gastrointestinal tract
5. Hepatic first pass effect and/or enterohepatic circulation resulting in some medicines not achieving the desired effect

Curcumin is an important active polyphenolic substance derived from turmeric, a plant of the ginger family [10]. The chemical structure of curcumin is shown in Figure 1. It has long been widely used as an edible natural pigment. Meanwhile, with the discovery of the chemical structure of curcumin (C_21_H_20_O_6_) as difluorocarbonyl methane in 1910, pharmacological studies on curcumin attracted extensive attention. In 1949, Schraufstatter et al. reported the antibacterial activity of curcumin [11], a finding that also drew widespread attention to its biological activity. In subsequent studies, curcumin has been successively found to have a variety of pharmacological effects, such as antitumor effects, protection against oxidative damage, and inflammatory responses [12–16]. Researchers have likewise conducted various studies on the pulmonary mechanism of action of curcumin and found that curcumin can inhibit A549 cell proliferation and enhance apoptosis by upregulating GUCY2GP, H2BFXP, LINC00623, and IncRNA, while downregulating IncRNA UCA1 [17–20]. Meanwhile, curcumin downregulates protein 66 homolog-collagen homolog (p66Shc), promotes the expression of RNA encoding SIRT1 histone deoxygenase, promotes protein autophagy, and inhibits ERS (endoplasmic reticulum stress), thereby reducing alveolar epithelial damage in COPD; on the other hand, it inhibits BEAS-2B cell proliferation and suppresses NF-*κ*B and COX-2 expression, thereby reducing airway inflammation and airway remodelling. It alleviates COPD symptoms in several ways and has a positive therapeutic effect. These studies imply that curcumin has great potential for clinical application in the treatment of pulmonary diseases, especially for COPD [21, 22].

However, the main drawback of curcumin is its poor solubility in water, which leads to low bioavailability [23]. Moreover, curcumin is readily hydrolyzed in neutral and alkaline environments [16, 24]. Therefore, it is necessary to design effective strategies to increase solubility and, most importantly, its bioavailability effectively. In conclusion, the advancement of these aforementioned properties has become key to the clinical application of curcumin.

A great deal of research in recent years has focused on improving the water solubility of curcumin. To date, researchers have offered a variety of solutions to this problem. Encapsulation of curcumin in a readily digestible lipid droplet to form a nanoemulsion delivery system is one effective approach [25]. Asli et al. prepared curcumin/cyclodextrin inclusion using the technology of electrospun nanofibrous webs, which improve the solubility of curcumin [26]. Undeniably, the abundance of nanoparticle techniques and methods did improve the water solubility and bioavailability of curcumin, but its nonnegligible that the complex preparation process hinders its widespread use and none of these formulations addressed the drug in terms of absorption and distribution, and none of them were suitable for pulmonary administration [27].

Our study proposes the application of spray drying technology to improve water solubility for the preparation of dry powder inhalers for pulmonary inhalation. Spray drying is a common drying technique used in traditional pharmaceutical production, and by adjusting its process parameters, the powder properties such as particle size, powder flow, and crystal morphology can be optimized [28, 29]. The aim of this study was to convert an ethanolic solution of curcumin into a solid dispersible powder with a particle size distribution suitable for pulmonary inhalation by spray drying to obtain an amorphous dried powder. According to available studies, amorphous drugs have a more disordered molecular structure and a higher energy state than crystalline drugs, and this state is more soluble, thus improving solubility and bioavailability [30]. Specifically, the current study showed that DPIs not only have ideal dispersion in the pulmonary, avoiding drug deposition, but also allow to control the particle size and inhaled dose of the drug in a precise range. They confirmed that DPIs have satisfactory absorption in the lungs and significantly improved bioavailability. These results provide important insights and support for further studies and applications of curcumin DPIs for COPD.

Mannitol is a naturally occurring six-carbon sugar alcohol that has a wide range of applications in the food and pharmaceutical industries due to its low metabolism and nonglycaemic index properties that make it less susceptible to oxidation in air. Mannitol is soluble in water and maintains good stability in aqueous solutions of acids/bases [31, 32]. In addition, it is soluble in glycerol, pyridine, and aniline, but slightly soluble in ethanol. Mannitol is also a highly effective dehydrating agent and osmotic diuretic, helping to minimise the risk of acute renal failure in renal transplant patients. Its pharmacological effects have also been demonstrated when inhaled into the lungs. Inhalation of mannitol produces an osmotic drive that allows water to enter the airway lumen while promoting effective coughing and stimulating mucociliary clearance, reducing mucus adhesion to the epithelium and promoting the binding of mucus and cilia, thereby increasing mucus clearance from the lungs [33]. Better pulmonary therapeutic effects can be achieved when formulated with curcumin as an inhaler. The principle of application and pharmacological action of the dry powder inhalation method of curcumin with mannitol as a carrier is shown in Figure 2.

In this research, different concentrations of curcumin ethanol solution were sprayed dry, and dry powder particles of different particle sizes were obtained, and their solubility and physical and chemical properties were further characterized by differential scanning calorimetry (DSC), Fourier transform infrared spectroscopy (FTIR), thermal gravimetric analysis (TGA), X-ray diffraction (XRD), and scanning electron microscopy (SEM). This work presents a novel curcumin-based DPI (drug powder inhalation) medicine for COPD (chronic obstructive pulmonary disease).

## 2. Materials and Chemicals

We chose analytical grade mannitol (≥99.8%) as the carrier for curcumin dry powder inhalation, which was purchased from Tianjin Beichen Founder Reagent Factory; curcumin (purity > 98.0%) was purchased from Tonghua Food Chemical Co.; the anhydrous ethanol (≥99.7%) used in the experiment was provided by Shanghai Titan Technology Co., Ltd.; the pure water used in this experiment was made by the laboratory.

### 2.1. Design of Experiments

According to the preliminary experiments and literature review, we learned that curcumin has low solubility in water and high solubility in ethanol; on the contrary, mannitol completes a good solvent in water and has low solubility in ethanol. In order to mix the two substances homogeneously and to achieve a similar and suitable particle size distribution, we had to dissolve both substances completely. We chose to use a mixture of anhydrous ethanol: water = 6 : 4 (v/v) as the dissolution medium.

Before starting the experiment, we added 5.0 g of curcumin to 3.0 L of anhydrous ethanol, sonicated it at 50.0 KHz for 10 min, and then stirred it well until it was all dissolved. Meanwhile, 45.0 g of mannitol was accurately weighed and added to 2.0 L of pure water, again, sonicated at 50.0 KHz for 10 min, and then stirred until dissolved. After the two solutions were configured, the aqueous mannitol solution was slowly poured along the glass plate into the ethanol solution of curcumin and mixed thoroughly to obtain 5.0 L of aqueous mannitol solution of curcumin at a mass concentration of 1.0% (m/v) (ethanol:water = 6 : 4 (v/v)).

In order to obtain products with a suitable particle size distribution (1–5 *μ*m), we took two initial solutions with a concentration of 1.0% and diluted them by adding different volumes of aqueous 60% ethanol to obtain 1.0 L of solutions with a mass concentration of 0.5% and 0.7%, and another 1.0 L of an initial solution with a mass concentration of 1.0% was accurately weighed under stirring to obtain 1.0 L of each of the three different concentrations. Stirring was carried out at the same rate under light-proof conditions.

After the experiments were started, the three solutions were fed with the same spray drying parameters and the spray dryer (Shanghai YC-015) was adjusted to the optimum parameters as follows: fan frequency 50.0 Hz, inlet air temperature 130.0 ± 1.0°C, outlet air temperature 127.0 ± 2.0°C, peristaltic pump speed 8.0 ml/min, spray pressure 0.40 MPa, and nozzle diameter 1.0 mm. Three spray-dried samples were obtained in the order of concentration, i.e., sample A (0.5%), sample B (0.7%), and sample C (1.0%).

### 2.2. Characterization of Samples

#### 2.2.1. UV-Visible Spectrophotometer (UV-Vis)

In order to investigate whether the spray drying process has a facilitating effect on the solubility of curcumin, we dissolved an excess of a physical mixture of curcumin and mannitol in water at room temperature, while an excess of the sample obtained by spray drying was dissolved in the same volume of water and sonicated at the same sonication frequency. The obtained suspension was centrifuged in a centrifuge tube at 4000 rpm/min for 20 min and the same volume of supernatant was diluted by the same multiple, respectively. Based on the characteristics of the absorption spectrum, we detected the absorption at wavelengths of 200–800 nm and plotted its UV absorption curve at 200–600 nm. The instrument used was a UV-2401 pc spectrophotometer, Shimadzu, Kyoto, Japan.

#### 2.2.2. Differential Scanning Calorimetry (DSC)

DSC analysis of raw materials and sample powders was performed using a differential scanning calorimeter (HSC-4 DSC, Henven, China). 8.0 g of the material to be analyzed was weighed precisely in a sealed aluminum pan, respectively, and encapsulated according to standard procedures. The powder was then heated to 300°C at 30°C with a heating rate of 5°C/min.

#### 2.2.3. Fourier Transform Infrared Spectroscopy (FTIR)

The raw materials and product samples used in the experiment were studied by Fourier transform infrared spectroscopy. Each sample was separately mixed with dried KBr powder and compressed into clear sheets at low humidity. A Thermo Fisher Scientific 6700 Fourier transform infrared spectrometer was used in the experiment.

#### 2.2.4. Microscope

In order to visually observe the morphology of the product particles, we observed the samples in a microscopic view (DFG-90DZ).

#### 2.2.5. Scanning Electron Microscope (SEM)

Place the lactose sample on a carbon strip on an aluminum sample needle. The gold-plated particles were observed at various magnifications using a JSM-7200F scanning electron microscope (SEM, JEOL Ltd.).

#### 2.2.6. Thermogravimetric Analyzer (TGA)

Samples were analyzed by thermogravimetric analyzer (TGA Q5000 V3.17 Build 265). Samples were tested in the instrument with N_2_ as balance gas and heat conduction gas, and the temperature was heated from 35.0°C to 350.0°C at a rising rate of 5.0°C per minute, and TGA curve was drawn based on the obtained heat flow data.

#### 2.2.7. N_2_ Absorption

The mesoporous adsorption experiments were performed on the powder samples to explore the pore size distribution in the samples and the relationship with the specific surface area and pore volume.

#### 2.2.8. X-Ray Diffraction (XRD)

XRD analysis was used to study the crystallization behavior of the samples. Solid samples were loaded on powder supports and analyzed using a Siemens D5000 diffractometer sample at a scan rate of 0.02 o/s, a scan current of 30.0 mA, and a scan voltage of 40.0 kV.

## 3. Results and Discussion

The novel curcumin-based DPI medicine is developed for COPD. During the dissolution process, a slow dissolution rate of curcumin crystals was observed. Under ultraviolet scanning (Figure 3), weak absorption was observed at 350–500 nm under physical mixing, with small absorption, indicating that the solubility of curcumin crystal in water at room temperature was low. However, the absorption of the sample after spray drying was significantly increased, and two obvious absorption peaks were observed in the range of 200–500 nm [34, 35]. The absorption peaks appear at 310 nm and 425 nm, respectively, probably indicating the shift in tautomers equilibrium from enol-keto to diketo tautomers [36]. Compared with the physical mixed solution, the absorption rate of the sample after spray drying was increased several times, proving that the spray drying process had a good dissolution promoting effect. In addition, the visible solids in the spray-dried sample mixture decreased significantly after 2 min during the dissolution process, indicating that the spray-dried samples had good solubility, which achieved not only excellent dissolution during inhalation but also prevented the spray-dried samples from dissolving too quickly to ensure delivery deep into the lungs for optimal therapeutic effect.

We carried out thermal analysis of the constituent materials in the experiment. By analysing the DSC curves of the samples (Figure 4), the maximum heat absorption peaks for curcumin and mannitol occurred at 196.2°C and 171.6°C, respectively. For the physical mixture, the heat uptake peak of mannitol shifted towards the high temperature region, with the maximum heat uptake occurring at 172.5°C, while the heat uptake peak of curcumin shifted to 184.4°C, which may be related to the slower heat transfer rate of the solid mixture. In the physical mixture, the heat absorption peaks of curcumin and mannitol were present simultaneously, while for the spray-dried samples, the overall heat absorption peak shifted towards the low temperature region, reaching 170.9°C; this may be attributed to differences in melting enthalpy due to polycrystalline formation. No significant heat absorption peaks were seen in samples A (0.5%) and B (0.7%), except for a very small heat absorption peak for curcumin visible in sample C (1%). This suggests that in samples A and B, curcumin has sufficient solubility at lower solution concentrations to be present mostly in the amorphous form after spray drying at the same temperature [37]. Apart from this, no significant differences were seen in the DSC curves of the three sets of samples.

Figure 5 showed the thermogravimetric curves of the three sets of samples in order from left to right. The three sets of samples show the same trend of weight loss as the temperature increases. These samples show excellent stability up to 225°C and do not show a trend towards weight loss until after 225°C, reaching a maximum rate at 325°C. The combined analysis of these three sets of samples showed that the physical composition of the spray-dried powders obtained from the different concentrations of solutions was essentially the same and all had excellent thermal stability.

The variation of peak intensity or wave number shift of the raw material, physical mixture, and spray driven samples was studied by FTIR (Figure 6). The absorption peak of that starting material curcumin and mannitol are present in the physical mixture at all wavelengths and the peaks of the physical mixture combine with the large vibration peaks of the respective starting material, e.g., the hydrogen and oxygen vibration peak at 3300–1 cm and the bands due to C–H in the plane bending vibration and C–C tensile vibration peaks in the range of 1300–1000^−1^ cm relative to the respective starting material, and many sharp bands of medium to weak intensity are observed in the figure. For the spray-dried samples, some sharp vibration peaks disappeared and combined into many flat weak-intensity vibration peaks, indicating that the hydrogen bond density and intensity were decreased, and the crystallinity was decreased [38]. However, for the 1000–1100^−1^ cm samples, the two vibration peaks were increased, which might be due to the increase of carbon-oxygen (C–O) vibration intensity under the low-density hydrogen bonds.

The size of curcumin-based DPI medicine is important for COPD treatment. Three groups of samples showed different sizes in the microscopic field of view. At the same magnification, the overall size distribution of the powder sample is positively correlated with the concentration. The higher the concentration is, the larger the average size is. A similar state was observed in the SEM field of view (Figure 7), where all three groups of samples exhibited smooth spherical surfaces, and again there was a significant positive correlation between size and solution concentration. However, the overall dimensions of all three groups of samples were in the range of 1–5 *μ*m, indicating that the powder obtained in the experiment performed an excellent aerodynamic effect when inhaled into the lungs at these solution concentrations. Interestingly, the size differences observed with SEM are not as large as they appear in the microscopic view, which may be due to the varying degrees of homogeneity of the dispersion. For similar samples in the porous state, nitrogen adsorption experiments were performed to calculate and evaluate the pore structure (Figure 8), whose porosity is visually represented by its BET adsorption and desorption curves. We plotted and analyzed its isotherm, BJH adsorption/desorption dV/log(w) pore volume, and BJH adsorption dA/log(w) area, respectively. The calculated average pore size was 8.38 nm. The pore volume for the width range of 1.7 ∼300 nm was 0.051327 cm/g. The BET surface area was 22.8439 m^2^/g. The large pore volume and surface area may provide better aerodynamic characteristics.

The X-ray diffractograms of the three sets of samples were also explored (Figure 9). The diffraction peaks for the mannitol polycrystalline form are marked in the black dashed box and that for curcumin in the red dashed box, with a possible overlap of the two substances in some parts. The results show that the crystal structures of the three groups of samples are not significantly different, while having a similar mannitol polycrystalline structure [39]. Some characteristic peaks of curcumin disappeared, for example, the two sharp diffraction peaks at 2*θ* = 9-10° disappeared and became short and flat, indicating that curcumin transformed into an amorphous structure [40, 41]. As the concentration of the solution increases, the diffraction peaks become sharp and steep, which may indicate a high amorphous content at low concentrations [41, 42]. Spray drying has been widely used in multiple drug carrying and delivery applications [43–45]. We think this work contributes to the pharmaceutical engineering.

## 4. Conclusion

Dry powder inhalation is one of the best ways to improve the efficiency of treatment of pulmonary diseases, or to improve the efficacy of diseases that cannot be treated by oral or intravenous administration. In this experiment, a dry powder inhalation of curcumin was prepared by spray drying technology, using mannitol as a carrier. On the premise of confirming its excellent pharmacological effect on COPD, mannitol and curcumin were sprayed together by spray drying technique to obtain a spherical powder with a particle size distribution of 1–5 *μ*m. The characterization results showed that the experimental product has good solubility and dissolution; its uniform spherical structure and appropriate particle size distribution can ensure that the DPI delivered deep into the lungs to achieve the best therapeutic effects, which provides a new idea for the treatment and prognosis of COPD.

## Figures and Tables

**Figure 1:** Chemical structure of curcumin.

**Figure 2:** Principles of application and pharmacological effects of dry powder inhalation of curcumin.

**Figure 3:** UV absorption curve of physical mixture and spray-dried sample at 200–600 nm.

**Figure 4:** DSC curves of spray-dried samples, raw materials, and physical mixture.

**Figure 5:** The TGA curves of the spray-dried samples A, B, and C (from left to right).

**Figure 6:** FTIR spectra of the raw materials, physical mixture, and samples.

**Figure 7:** Micrographs of three groups of samples.

**Figure 8:** SEM images of the sample A (A1, A2), sample B (B1, B2), and sample C (C1, C2) (5000x (left) and 2000x (right), respectively).

**Figure 9:** X-ray diffraction patterns of three groups of samples.

## Data Availability

All data supporting this work are included within the paper.
